# Application of Multimodal Neuroimaging in the Treatment of Neurological Patients

This article has been retracted.

**DOI:** 10.1155/2022/5502213

**Published:** 2022-05-02

**Authors:** Lixia Zhang, Guiyang Li, Lunzhong Zhang

**Affiliations:** Encephalopathy Department of Weifang Hospital of Traditional Chinese Medicine, China

## Abstract

**Objective:**

In order to study the application of multimodal neuroimaging in the treatment of neurological patients, the brain of patients was scanned and identified through multimodal neuroimaging, so as to provide basis for doctors to judge their diseases and give treatment plans.

**Method:**

Understand the principle of multimodal neural scene currently used through literature analysis, analyze the current level of neurological diseases in the medical field and the application of multimodal neural image in diseases, recalculate the imaging examination data through neurofuzzy algorithm, and obtain a more optimized identification method than the previous visual judgment method.

**Result:**

The image inspection data is dimensioned through computer spatial convolution. At this time, the output two-dimensional array is not accurate enough. It needs to be processed again through fuzzy spatial convolution to obtain relatively accurate data output, generate a small two-dimensional array, and use the convolution core for the spatial convolution process of two-dimensional array. The algorithm uses neural network machine learning algorithm to identify and judge the inspection data.

**Conclusion:**

Through this algorithm to identify the examination data, the early diagnosis sensitivity of intracranial space occupying lesions and intracranial hematogenous lesions are more than 20% higher than the previous traditional recognition methods, which provides a medical imaging basis for the early diagnosis and treatment of acoustic diseases, and improves the treatment probability and prognosis quality of life of neurological patients.

## 1. Introduction

In the imaging examination related to neurosurgery, subject to the physical principle of imaging, based on electromagnetic, infrared, and other examination methods, it is difficult to effectively determine the early lesions by using a single imaging examination method. Even if multiple examination methods are used together, it is difficult to obtain effective results in the interpretation of imaging examination results. Therefore, in the early treatment of neurological patients, there are problems of difficult examination and diagnosis, which leads to the general course of disease that has developed to the middle and late stage when patients with intracranial lesions are diagnosed.

In the technical system reported in relevant literature, using the existing intracranial imaging examination means and deep data mining algorithms such as machine learning algorithm, the data of multiple imaging examination results are fused to form a multimodal neuroimaging examination system. The system does not change the traditional examination system, does not upgrade the intracranial imaging examination hardware system, mounts the data analysis host outside the intracranial imaging examination system, and realizes multimodal data fusion and deep data mining.

This study uses the literature analysis method to summarize the technical path and relevant data in the relevant literature and explore the application path and effect of multimodal neuroimaging in the early diagnosis of patients with intracranial nervous system diseases.

## 2. Available Resources for Neuroimaging Techniques

EEG is based on electromagnetic signal detection (electroencephalography EEG) 和 magnetoencephalogram (magnetoencephalography, MEG). It is a technical means to explore the physiological structure of the brain. Because it is not affected by the external physical structure of the head layer, it has high recognition of the internal space of the head, and the data collection time is short. It is more suitable for the detection of children.

Dian and Lingzhi (2021) pointed out that childhood autism spectrum disorder (ASD) is an abnormal phenomenon characterized by language cognitive difficulties and uncontrolled behavior, which is considered to be a disease with limited neurodevelopment. The timely discovery of ASD can improve children's cognitive development and normal language development through scientific intervention. Therefore, the early diagnosis of ASD is particularly important. This study discusses the brain image characteristics of ASD through the advantages of EEG and MEG in identifying the early symptoms of ASD, so as to provide a basis for the early diagnosis of ASD [1]. Electromagnetic signal detection EEG is mainly used to record patients' brain waves to analyze the types and changes of brain waves to assist in the diagnosis of diseases, especially for the diagnosis of complex causes.

Language is not only a natural instinct of human beings but also a feature of human civilization. Language is made after thinking through the brain, these sounds are the result of brain activity, and they have strong logic and subjectivity. Pan et al. (2019) pointed out that speech is the cognitive behavior after brain activity. How the brain organizes speech symbols and forms language expression behavior through dynamic activities has aroused the exploration of the brain in the field of neuroscience. The technology based on brain imaging appears, and the effect of speech nerve function on speech is found through its tracking research, which provides a basis for studying how the brain works continuously on speech [2].

Functional magnetic resonance imaging (fMRI) is based on blood oxygen level dependent measurement. It is mainly through magnetic resonance imaging to detect the activity track of neurons and its influence on blood. Based on the convenience of fMRI, there is no radiation exposure problem and the activity track of real-time signal transmission. As a result, it has been widely used in the field of brain functional imaging since its emergence, mainly in the research of brain and spinal cord. Qin et al. (2021) believe that the brain is one of the more important organs of human beings. People have never stopped the research on brain function and accurately locate the brain activity area through non-invasive means. It is pointed out that OSAHS (obstructive sleep apnea hypopnea syndrome) is caused by apnea and poor breathing during sleep, accompanied by the decrease of blood oxygen saturation, which will lead to serious brain death. This study analyzed the course of OSAHS by detecting the changes of cerebral blood flow, focusing on the principle and application of fMRI [3].

Brain tumors can occur in three age stages, mainly in the middle-aged and elderly population, and the cause of the disease has not been determined. Clinically, it is considered that the pathogenesis of tumors is related to many factors such as genetics and environment, which is generally divided into malignant tumors and benign tumors. Weimin (2016) based on the current medical level, both malignant and benign tumors will cause brain function damage to the affected brain parts and even endanger life safety. The tumors with different lesions will have different clinical treatment schemes. Therefore, the location, nature, size, development direction of the tumor, and the degree of invasion to the surrounding tissues are studied, and the corresponding diagnosis is given. The choice of treatment scheme is particularly important for the recovery of the disease. In this paper, brain function imaging is used to diagnose brain tumors completely, so as to assist doctors in the selection of treatment scheme in follow-up treatment, and detects the most active cell structure in tumors [4].

Near infrared spectroscopy (NIRS) technology based on metabolic level measurement is to scan the deep tissue of bone by using the penetration of infrared spectroscopy technology. Because infrared spectroscopy technology not only has the characteristics of convenience, efficiency, accuracy, and low cost but also has the advantages of no intervention, no consumption of chemical reagents, and no pollution in the application of scanning bone imaging, this technology has been popularized and applied to various adjuvant treatments in the medical field in recent years. Bao (2021) pointed out that the application of near-infrared spectroscopy in brain tissue oxygen monitoring equipment generally monitors the oxygen saturation during surgery and intensive care. The near-infrared tissue oxygen monitoring equipment can continuously and in real time monitor the brain oxygen parameters without intervention, which has been popularized and applied in cognitive neuroscience and mental diseases [5].

## 3. Fusion Algorithm of Multimodal Imaging Examination Data

Multimodal medical image fusion provides auxiliary diagnostic basis for clinical diagnosis through the combination of computer, biological science, and medical technology. It integrates medical image processing technology and medical impact diagnosis technology. And only when multiple image data are integrated into one image data can it be called fusion. The result is to optimize the information resources from many different sources and finally get more useful information sources than any one.

According to the characteristics of medical image fusion, Wen et al. (2017) analyzed the widely used medical image fusion technology, carried out simulation experiments in MATLAB environment, and provided reference data for relevant medical fields [6].

In this algorithm, each two-dimensional array is de dimensioned by the linear space convolution method to obtain a two-dimensional array. At this time, the two-dimensional array is not significant enough. It needs fuzzy space convolution to obtain an accurate two-dimensional array. After iterative processing, a more reliable processed image is finally obtained. The above logical architecture is shown in Figure 1.

The statistical significance of results spatial convolution algorithm is to perform specific information enhancement operations on the two-dimensional array of specific neuroimaging examination images, such as edge enhancement, peak enhancement, etc., and its basis function is as shown in formula (1):

(1) $$\begin{array}{c} F_{i}\left(x,y\right)=\int_{-\infty }^{+\infty }g\left(t\right)S_{i}\left(x-t,y-t\right). \end{array}$$

Among *g*(*t*)  is convolution kernel, *S*_*i*_ is the convoluted two-dimensional array, *t* is convolution pointer, *F*_*i*_(*x*, *y*) is the convoluted output two-dimensional array, and *i* is the data source number of the convoluted image. The convolution process does not change the image scale before and after convolution; that is, a two-dimensional array processed in a specific enhancement direction is generated for a specific two-dimensional array, such as edge enhancement and peak enhancement;

The statistical significance of the fuzzy space convolution algorithm is to realize data fusion of multiple two-dimensional arrays of neuroimaging examination images. The basis function is as follows (2):

(2) $$\begin{array}{c} \text{G}\left(x,y\right)=\overset{n}{\underset{i=1}{\sum }}\overset{5}{\underset{j=0}{\sum }}A_{i,j}S_{i}{\left(x,y\right)}^{j}, \end{array}$$

among which *n* is the number of input two-dimensional arrays, *j* is the order of polynomial for fuzzy convolution, *A*_*i*,*j*_ is the coefficient to be regressed of the *i*-th image in the *j*-th order polynomial, *S*_*i*_(*x*, *y*) is the *i*-th input 2D array, and *G*(*x*, *y*) is the two-dimensional array output after convolution. In general mode, for a total of NA_*i*,*j*_, there is a numerical relationship of *A*_1,*j*_ = *A*_2,*j*_ = ⋯ = *A*_*n*,*j*._

The convolution kernel used in the spatial convolution process of two-dimensional array, such as *g*(*t*), used in formula (2) above, is a small two-dimensional array, and its generation algorithm also uses the neural network machine learning algorithm, as shown in Figure 2.

In Figure 2, the fuzzy neural network (FNN) uses the sixth order polynomial depth iterative regression node basis function, as shown in formula (3). A multicolumn neural network is used to generate the values of each element of the convolution kernel. Each column adopts log depth iterative regression neural network (lnn), and its basis function is as shown in formula (4).

If the fuzzy neural network is used to control the recent change law of time series data, or the minimum number of nodes is needed to realize the fuzzy convolution of data, the sixth-order polynomial depth iterative regression basis function with complex function curve and rich regression coefficients needs to be used, and its expression is shown in formula (3):

(3) $$\begin{array}{c} y=\overset{n}{\underset{i=1}{\sum }}\overset{5}{\underset{j=0}{\sum }}A_{j}x_{i}^{j}, \end{array}$$

Among which *A*_*j*_ is the coefficient to be regressed of the *j*-th order polynomial; that is, each node in the formula contains 6 coefficients to be regressed from *A*_0_ to *A*_5_; *j* is polynomial order. The meanings of other mathematical symbols are the same as those above.

The basis function of log depth iterative regression neural network module is shown in formula (4):

(4) $$\begin{array}{c} y=\overset{n}{\underset{i=1}{\sum }}\left(A∙\log x_{i}+B\right), \end{array}$$

among which *A* and *B* are coefficients to be regressed. The meanings of other mathematical symbols are the same as those above.

## 4. Hardware Technology of Multimodal Neuroimaging Fusion Data

According to the above research on the algorithm of multimodal neuroimaging inspection fusion data, the software part of multimodal neuroimaging inspection can be determined, and the hardware technology of multimodal neuroimaging inspection fusion data must reach a certain degree to meet the inspection requirements. The hardware technology of multimodal neuroimaging fusion data must be combined with the current Internet environment [7, 8]. The data logic diagram of the bus system of a single host is shown in Figure 3 below;

The hardware technology needs to use a single host to complete the functions of data management, floating-point computing, and machine learning. These three hardware technologies are the mainstream technology path of multimodal neuroimaging fusion data. Among them, floating-point calculation is real number operation, but the computer can only store integers; so, the real numbers obtained by floating-point operation are divisors. The data analysis host uses high-speed and large capacity dynamic storage (RAM) technology, multithreaded and multicolumn workstation technology, multithreaded and multicolumn floating-point computing unit (GPU) management technology, redundant arrays of independent disks (RAID), etc.

In Figure 3, PCI EBUS is connected to multiple GPU devices, each GPU device is equipped with independent ram, and raid is connected to multiple HDDs. Until the data capacity can meet the data mining requirements, South Bridge is connected with an *s*-nid to connect to the main switch of outpatient hospital system, and the other South Bridge is connected with an *m*-nid neuroimaging device to collect the information of all neuroimaging devices. At present, the host system allows up to two rows of CPUs to access, and each row of CPUs is equipped with independent ram. Although the price of this device is relatively expensive, however, a single host device can be used to meet the requirements of data mining.

## 5. Diagnostic Sensitivity Statistics in Relevant Literature

At present, with the development of global information technology and its application, medical imaging has become an indispensable and important link of modern medical technology, which greatly increases the diagnosis effect of diseases, saves medical costs, and increases the treatment probability of patients. This paper analyzes and reviews the diagnostic sensitivity of multimodal neuroimaging in the past and uses statistical methods to count the early diagnostic sensitivity of intracranial space occupying lesions and intracranial hematogenous lesions in neurological patients.

### 5.1. Sensitivity of Early Diagnosis of Intracranial Space Occupying Lesions

Intracranial space occupying lesions are the general name of a group of diseases occupying a certain space in the skull cavity. The common diseases are intracranial tumors, intracranial hemorrhage, and brain abscess. This paper reviews and analyzes the causes of cysts, hemangiomas, connective tumors, and cancer in the relevant literature and counts the early diagnostic sensitivity data of their separate examination and multimodal examination, as shown in Table 1 below.

In Table 1, it is obvious that the early diagnosis sensitivity of multimodal examination is higher than that of single examination, and the precondition for the treatment of intracranial lesions is accurate diagnosis and accurate positioning. Therefore, the use of multimodal examination can improve the treatment effect of such patients. In order to more clearly compare the difference of early diagnosis sensitivity between separate examination and multimodal examination, Figure 4 is made according to the statistical data in Table 1.

It can be seen more clearly from Figure 4 that the early diagnosis sensitivity data of the two examination methods are different. The early diagnosis sensitivity of single examination for different causes is about 75%, while the early diagnosis sensitivity of multimodal examination is about 95%. The early diagnosis sensitivity of multimodal examination is about 20% higher than that of single examination, which is a leap forward. This will provide a more favorable basis for the diagnosis and treatment of patients with intracranial space occupying lesions.

### 5.2. Sensitivity of Early Diagnosis of Intracranial Hematogenous Lesions

Intracranial hematogenous lesions, also known as intracranial hemorrhagic lesions, refer to lesions caused by intracranial hemorrhage or hematoma formation, or hemorrhagic stroke changes of original lesions. Generally, it can be divided into spontaneous intracranial hemorrhage and traumatic intracranial hemorrhage. Spontaneous intracranial hemorrhage includes hemorrhage or hematoma formation after vascular malformation rupture, hypertensive intracerebral hemorrhage, tumor stroke, and some unexplained intracranial hemorrhage. The early diagnosis sensitivity of intracranial hematogenous diseases counted in this paper is arteriosclerosis, spasm, ischemic stroke, and hemorrhagic stroke. The early diagnosis sensitivity data of the two examination methods are shown in Table 2 below.

In Table 2, the comparison of early diagnosis sensitivity data between the two examination methods has significant statistical difference (*P* < 0.05). The early diagnosis sensitivity of multimodal examination is much higher than that of single examination, and the early diagnosis sensitivity data of multimodal examination with different etiology are more than 95%, while the early diagnosis sensitivity data of single examination are only about 75%. In order to facilitate readers to more clearly understand the difference of sensitivity data of the two examination methods for early diagnosis of intracranial hematogenous lesions, Figure 5 is made according to Table 2 above.

In Figure 5, it can be clearly seen that the sensitivity data of multimodal examination for early diagnosis of intracranial hematogenous lesions of different etiologies are much higher than that of single examination. The early diagnostic sensitivity of multimodal examination is more than 15% higher than that of single examination, which not only increases the diagnostic accuracy of intracranial hematogenous lesions but also provides a more favorable basis for the follow-up treatment of patients.

According to the early diagnosis sensitivity data in Tables 1 and 2, Table 3 is obtained. The data in Table 3 is the difference between multimodal examination and separate examination of intracranial space occupying and hematogenous lesions.

It can be seen from Table 3 that the sensitivity of multimodal imaging examination technology for early diagnosis of different causes of intracranial space occupying lesions and intracranial hematogenous lesions is about 20% higher than that of single examination technology, which greatly increases the accuracy of early diagnosis of neurological patients and the evaluation value for the formulation of treatment plan.  Figure 6 is the histogram of the data in Table 3. It is convenient for readers to better see the regularity of the data.

In Figure 6, it can be seen that the difference range of early diagnosis sensitivity between multimodal examination and separate examination of intracranial space occupying lesions and intracranial hematogenous lesions is about 20%.

## 6. Application Prospect of Multimodal Neuroimaging Technology in the Treatment of Neurological Patients

The treatment of neurological patients is mostly carried out through surgery, and the brain nerves are complex. If you are not careful, there will be serious consequences. Multimodal neuroimaging images provide doctors with brain morphology scanning to judge the condition of lesions through empirical identification. As the imaging technology is relatively mature, it can complement each other according to its advantages. The more common clinical multimodal imaging technology is to carry out multiple imaging analysis of multimodal imaging technology to comprehensively understand the patient's lesion, so as to make a more accurate judgment and give the best treatment scheme.

The best way to accurately remove lesions during operation is to use multimodal imaging combination technology to conduct comprehensive physical examination of patients, fuse and analyze the image data of various functional lesions, so as to accurately find the diseased tissue and select the best surgical scheme suitable for patients, remove the diseased tissue to the greatest extent, and protect the brain nerve function, so that the patient can get the optimal treatment. Mingming and Junfeng (2021) take medulloblastoma as an example, and the conventional treatment method is the combination of pathology and molecular diagnosis. Based on the emergence of imaging omics, it provides a new direction for its noninvasive identification of medulloblastoma subtypes. This study discusses and analyzes the application of multimode imaging technology in children's medulloblastoma [9]. Meng (2021) analyzed the multimodal neuroimaging study of senile depression. He said that the systematic collection of multimodal data such as resting state functional MRI (RS fMRI), structural MRI (SMR I), and clinical neurological scale data can provide a basis for finding neuroimaging markers for patients [10]. The first mock exam is the first mock exam. The application of multimodality neuroimaging technology can make up for the deficiency of single modal. Xiangyuan (2019) analyzed the research and application of new multimodal neuroimaging technology, saying that the development of new neuroimaging technology is an important driving force for the development of brain science, and neuroimaging research belongs to a typical interdisciplinary subject. Researchers need solid multidisciplinary background knowledge and systematic in-depth learning and training to make achievements in this field [11]. Dongsheng (2020) analyzed the research of multimodal neuroimaging in the treatment of refractory depressive disorder and believed that the application of multimodal neuroimaging can effectively help patients recover in advance [12, 13].

In the field of neuromedicine, technological reform will bring qualitative changes in treatment results. The application of assistive technology guides clinical diagnosis and treatment. Nowadays, the combination of various medical imaging technologies and high technology is changing the diagnosis and treatment methods of patients with neuropathy. Through the cognition of Daji's functional structure, people gradually pay attention to the relationship between neuropathy and brain nerve function.

## 7. Summary

With the continuous promotion of neuroscience and information science, neuroimaging has also made great progress, which can make human beings better carry out noninvasive inspection, observation, and recording of living bodies. Gao (2022) studied the research progress and practical application of multimodal neuroimaging technology. With the rapid development of neuroimaging technology and related data processing methods, multimodal neuroimaging fusion is widely used in neuroscience, clinical diseases, and other research fields [14]. This study uses the literature analysis method to analyze the multimodal imaging technology. Multimodal imaging is of great significance in the early diagnosis of neurological patients. It can accurately judge the changes in the complexity of brain microstructure and provide a basis for the customization of follow-up individualized treatment plan, course monitoring dynamic observation, and postoperative prognosis evaluation that provide medical imaging basis. Multimodal neuroimaging technology can be applied to clinical medical imaging examination as the neuroimaging detection index of neurological patients, so as to provide a more favorable image basis for accurate diagnosis and follow-up treatment of neurological patients. In the follow-up, we will further explore the role of multimodal neuroimaging technology in the treatment of neurological patients and widely apply this technology to the treatment of neurological patients.

## Figures and Tables

**Figure 1:** 2D array fusion algorithm for neuroimaging examination.

**Figure 2:** Convolution kernel generation algorithm for multimodal neuroimaging.

**Figure 3:** Data logic diagram of bus system of single host.

**Figure 4:** Comparison of early diagnostic sensitivity of intracranial space occupying lesions.

**Figure 5:** Comparison of early diagnostic sensitivity of intracranial hematogenous lesions.

**Figure 6:** Comparison of early diagnosis sensitivity difference between multimodal examination and separate examination.

**Table 1:** Comparison of early diagnostic sensitivity of intracranial space occupying lesions.

Inspection classification	Cyst (%)	Hemangioma (%)	Connective tumor (%)	Cancer (%)	Comprehensive (%)
Separate inspection	76.41	73.51	74.39	75.18	74.35
Multimodal inspection	95.78	96.67	95.75	94.68	94.57
*t*	3.654	3.587	3.246	3.127	3.572
*P*	0.026	0.023	0.019	0.016	0.021

**Table 2:** Comparison of early diagnostic sensitivity of intracranial hematogenous lesions.

Inspection classification	Arteriosclerosis (%)	Spasm (%)	Ischemic stroke (%)	Hemorrhagic stroke (%)	Comprehensive (%)
Separate inspection	73.68	76.21	77.28	76.91	75.51
Multimodal inspection	96.38	97.28	96.17	95.82	96.34
*t*	4.386	4.284	4.124	4.394	4.235
*P*	0.035	0.031	0.025	0.033	0.028

**Table 3:** Comparison of sensitivity difference between multimodal examination and single examination in early diagnosis of intracranial lesions.

Intracranial space occupying lesions	Cyst (%)	Hemangioma (%)	Connective tumor (%)	Cancer (%)	Comprehensive (%)
	19.37	23.16	21.36	19.5	20.22
Intracranial hematogenous lesions	Arteriosclerosis (%)	Spasm (%)	Ischemic stroke (%)	Hemorrhagic stroke (%)	Comprehensive (%)
	22.7	21.07	18.89	18.91	20.83

## Data Availability

The data underlying the results presented in the study are available within the manuscript.

## References

[1] Dian X., Lingzhi K. (2021). Early screening and diagnostic indicators of autism spectrum disorders based on magnetoencephalogram. *Chinese Journal of hearing and language rehabilitation*.

[2] Pan Y., Jiajie Z., Peiqing J., Nai D. (2019). Neural coding of continuous speech -- Research Progress of EEG and magnetoencephalogram. *Journal of physiology*.

[3] Qin W., Guangbin C., Feng A., Zili Z., Sheng L., Yanxi X. (2021). Brain dysfunction and its mechanism in patients with OSAHS: based on RS fMRI degree centrality method. *Radiology practice*.

[4] Weimin W. (2016). Application value of functional magnetic resonance imaging in the diagnosis of brain tumors. *Abstract of the world's latest medical information*.

[5] Bao C., Yao H., Wang Y., Zhijian Z., Quanfu W., Xia W. (2021). Research progress of brain oxygen detection system based on near infrared spectroscopy. *Sensors and Microsystems*.

[6] Wen C., Yu Y., Meihong Z. (2017). Simulation of multimodal medical image fusion based on MATLAB. *Electronic technology and software engineering*.

[7] Jing C. (2021). Construction of hospital image resource information system under Internet plus medical treatment. *China new technology and new products*.

[8] Ming Q., Xiaofen W. (2017). Using internet technology to improve the examination process of radiology patients. *China Medical equipment*.

[9] Mingming Z., Junfeng W. (2021). Research progress of multimodal imaging technology using optic nerve sheath diameter to monitor intracranial pressure. *Journal of clinical and pathology*.

[10] Meng D. (2021). Multimodal neuroimaging study of senile depression. *University of Electronic Science and technology*.

[11] Xiangyuan D. (2019). Training course on scientific research and application of new multimodal neuroimaging technology. *Radiology practice*.

[12] Dongsheng L. V. (2020). Multimodal neuroimaging study of modified electroconvulsive therapy in the treatment of refractory depressive disorder Inner Mongolia Autonomous Region. *mental health center of Inner Mongolia Autonomous Region*.

[13] Gao P. (2022). Li Haifang Research progress and practical application of multimodal neuroimaging technology. *Journal of Taiyuan University of Technology*.

[14] Fei T., Linling L., Mengying W. (2019). Multimodal neuroimaging fusion method and its application in diagnosis and treatment of brain diseases. *International Journal of Biomedical Engineering*.

